# The Research Progress in the Application of Ceramic Nanofibers in Antibacterial Textile Materials

This article has been retracted.

**DOI:** 10.1155/2022/9910266

**Published:** 2022-11-08

**Authors:** Miaoqing Xi, Xiaoming Yang

**Affiliations:** Donghua University, Shanghai 200051, China

## Abstract

In order to investigate the application effect of ceramic nanofibers in antibacterial textile materials and improve the comprehensive use efficiency of antibacterial textile materials, ceramic nanofibers were introduced firstly and their fabrication methods and specific functions were discussed. Then, the antibacterial textile materials were introduced and their main uses and contributions were discussed. Finally, the application of ceramic nanofibers in antibacterial textile materials was investigated based on CiteSpace software. The results showed that the research on ceramic nanofibers had increased rapidly since 2000. Also, the number of the foreign literature retrieval was about 9,200 at most and 6,300 at least. The number of Chinese literature was about 6,000 at most and 1,000 at least. It can be seen that the current research of ceramic nanofibers is quite mature. But the quantity of the research on ceramic nanofibers in the application of antibacterial materials is relatively small. In the foreign literature retrieval, the number of the literature was about 1,300 at most and about 220 at least. In the Chinese literature retrieval, the number of the literature was about 600 at most and about 30 at least. It can be seen that the current domestic research on the application of ceramic nanofibers in antibacterial textile materials is not mature, but the foreign research is relatively good. The research not only provides a reference for the further research of ceramic nanofibers but also contributes to the improvement of antibacterial textile materials.

## 1. Introduction

At present, with the continuous progress of society and the continuous improvement of people's living standards, textiles not only meet people's basic dressing needs but also are used in outdoor sports equipment, special professional work clothing, wearable electronic clothing, and other fields. The specific meaning of functional textiles refers to as follows: in addition to its basic textile properties, textiles also have the following functions: antibacterial, anti-electromagnetic radiation, anti-mildew, anti-mite, anti-water, anti-oil, anti-mosquito, anti-moth, anti-wrinkle, anti-ironing, anti-ultraviolet, antiviral negative ion health care, infrared physical therapy, and magnetic therapy [1, 2]. The development of functional textiles integrating multiple functions greatly optimizes the development value of traditional textiles and greatly expands the application field, which has broad market prospects and practical value. As a kind of high-quality lightweight material, ceramic nanofibers are synthesized in a simple and fast way. Therefore, it is an important research to use it as the basic material of antibacterial textile materials and exert its antibacterial properties through the synthesis technology [3]. Although the research is not mature, there are many research studies providing reference for it.

Fu et al. reviewed the research progress of ceramic nanofiber materials from the perspectives of carbides, nitride, and oxides, reported a new method for the preparation of SnO_2_ nanofiber—thermal explosion deformation synthesis method, and discussed the basic conditions for the preparation of SnO_2_ nanofiber by this method. SnO_2_ nanofibers were prepared by thermal explosion deformation synthesis and the data were analyzed. The results showed that the diameter of the SnO_2_ fiber was about 20∼100 nm and the X-ray diffraction spectrum of the SnO_2_ fiber was consistent with that of the standard SnO_2_ fiber. Therefore, compared with other methods, the thermal explosion deformation synthesis method had the advantages of simple equipment, convenient operation, high productivity, and no caking of products. Short fibers of different lengths were obtained by slight extrusion [4]. Chen et al. used the halo method to determine the dissolution types of 12 kinds of textiles. The results showed that antibacterial bandwidths of sample No. 1 used for the test of *Escherichia coli* and *Staphylococcus aureus* were 2.0 mm and 1.5 mm, respectively. All the other 11 textiles had antimicrobial bandwidth of less than 1.0 mm and were considered insoluble. On the other hand, the antibacterial performance of 12 kinds of textiles was quantitatively evaluated by the vibration method. The results showed that the antibacterial rate of sample 1 against *Escherichia coli* of material 2 was superior to that of material 1. In the four non-antibacterial samples, the antibacterial rate of the other nine fibers against *Staphylococcus aureus* was higher than that against *Escherichia coli*. Therefore, it was speculated that the type of fiber antibacterial finishing agent and fiber dyeing or finishing process had an impact on the bacteriostatic rate [5]. Koyuturk and Soyaslan pointed out that composite materials with antibacterial function had the ability to inhibit and kill microorganisms and could inhibit the growth of microorganisms and reduce the damage caused by microbial invasion. Antibacterial materials and products could be obtained by mixing ordinary materials with antibacterial agents with the help of surface treatment techniques, which exhibited microbial inhibition through surface contact antibacterial mechanisms. Organic-inorganic antibacterial agent and inorganic antibacterial agent were important components in antibacterial materials. Organic-inorganic compound antibacterial agent and nanoscale antibacterial agent are the developing directions of antibacterial agent in the future. Applicable antibacterial function composite materials mainly included antibacterial plastics, antibacterial fiber cloth, antibacterial ceramics, antibacterial coatings, antibacterial stainless steel, and so on. Antibacterial composite materials and products created new opportunities for energy conservation and emission reduction [6]. Raza et al. proposed a nano-ceramic antibacterial coating, which was calculated according to the weight of the antibacterial coating design number, including the following components: 30∼45 parts of siloxane, 6∼12 parts of water-based alkyd resin emulsion, 5∼10 parts of antibacterial nanoparticles, 8∼16 parts of potassium titanate whiskers, 5∼10 parts of nano-ceramic powder, 12∼18 parts of nano-perlite, 3∼6 parts of alumina fiber, 1∼3 parts of dispersant, 1∼3 parts of thickening agent, 0.2∼1 part of defoamant, and 15∼25 parts of water. The nano-ceramic powder was mainly prepared by nano-zirconia, nano-silicon carbide, nano-titanium nitride, and nano-zinc oxide. The antibacterial nanoparticles were a mixture of silver nanoparticles and titanium dioxide nanoparticles. The coating not only had excellent antibacterial performance but also had good high temperature resistance [7].

Based on the above, in the research, the characteristics of ceramic nanofibers were discussed first. Then, the basic properties of antibacterial textile materials were discussed. Finally, CiteSpace software was used to describe the application of nano-ceramic fibers in antibacterial textile materials. The research not only provides a reference for the application of ceramic nanofibers but also contributes to the comprehensive optimization of antibacterial textile materials.

## 2. Research Theories and Methods

### 2.1. Ceramic Nanofibers

Ceramic material is a kind of research frontier and hot material in the field of materials. It is very light in weight and has very good stability at high temperature as well as excellent mechanical strength and corrosion resistance. The use of ceramic materials has a long history. Since ancient times, ceramic materials have been used in many fields, including photoelectric, sensor, protective material, catalyst carrier, drug carrier, and so on [8].

The existence of the fiber material is very common, which is widely distributed in nature. It first appeared in the process of spiders making the web by using protein liquid, about more than 1 million years ago. Also, in nature, other creatures can also make fiber materials by their own characteristics. So, ancient people obtained fiber materials in nature by raising silkworms, picking cotton, and using other ways and processed synthetic fiber materials, which are used in a variety of fields. At the same time, with the continuous development of human industrial skills, chemical production technology is more and more mature. So, humans successfully prepared the chemical synthetic fiber. In addition, from the ancient silk woven fiber to the modern synthetic fabric fiber, to the current organic, inorganic, and nanofiber, the application of fiber materials has always been one of the main research fields in materials science, chemistry, biomedicine, and other disciplines [9]. Among them, nanomaterials usually refer to the micromaterials with the diameter of 1–100 nanometers. Also, the application methods and application effects of nanomaterials in different disciplines are very different, so there are many preparation methods [10, 11]. Among them, the electrostatic spinning technology is an advanced method to prepare nanometer fiber materials. The main advantage of the electrostatic spinning technology is that it can directly and continuously prepare nanofiber materials, so the development and application prospect of the electrostatic spinning technology is very broad. Similarly, the electrostatic spinning technology also has a strong advantage in the preparation of ceramic nanomaterials, so it has become a research focus in the preparation of ceramic nanofibers. Ceramic nanofibers mainly refer to the nanofibers in 1 micron in diameter. The physical and chemical properties of the ceramic nanofibers are extremely outstanding. At the same time, it also can be made for membrane material. So, the ceramic nanofibers are widely used in energy storage, electrochemical, photoelectric materials, environmental engineering, catalytic industry, and other fields [12].  Figure 1 shows the main design of the electrostatic spinning technology.

As shown in Figure 1, the electrostatic spinning technology is the main method for preparing ceramic nanofibers, which can be prepared as membrane materials. Then, ceramic nanofiber membranes can be applied in a variety of fields through the synthesis technology, so the development prospect of ceramic nanofiber materials is very broad [13]. When the electrostatic textile technology is calculated, the calculation formula is as follows.

(1) $$\begin{array}{c} L=\frac{4KQ^{3}}{\pi \rho^{2}I^{2}}\left(\frac{1}{R_{0}^{2}}-\frac{1}{r_{0}^{2}}\right),\\ R_{0}={\left(\frac{2\sigma Q}{K\pi \rho E}\right)}^{1/3}, \end{array}$$

where *Q* represents the flow rate of the original liquid; *K* represents the conductivity of the original liquid droplet; *E* represents the electric field intensity; *ρ* represents the density of the original liquid; *r*_0_ represents the initial radius of the original liquid droplet; and *I* represents the current intensity through the original liquid droplet [14]. Because of the instability in the preparation process, the radius of the droplet can also be calculated, and the calculation formula is as follows.

(2) $$\begin{array}{c} r\left(Z\right)={\left(\frac{\rho Q^{3}}{2IE\pi^{2}}\right)}^{1/4}Z^{-1/4}, \end{array}$$

where *Z* is the number of droplets.  Table 1 shows the main raw materials for preparing ceramic nanofiber materials by the electrostatic spinning technology [15].

As shown in Table 1, the research mainly investigated the application of ceramic nanofibers in antibacterial textile materials through CiteSpace, so as to determine the development status of ceramic nanofibers.

### 2.2. Antibacterial Textile Materials

Antibacterial materials emerged at the end of the 20th century, and its development speed is very fast. From the beginning of its rise, it has become a research hotspot in the field of materials and rapidly developed into a new type of functional materials, mainly with the function of killing microorganisms on its surface independently. With the development of society, people have higher and higher requirements for living standards and health, so the demand for antibacterial materials in human society is also increasing. Also, antibacterial materials have been widely used in building materials, construction, communication, home appliances, packaging, and other fields [16]. Textiles are the most commonly used material for human beings. In the process of contact with them, human sweat, sebum, and other secretions are excellent sources of nutrition for various microorganisms. In the appropriate external conditions (including humidity, temperature, and so on), microorganisms grow and reproduce rapidly and spread diseases in a variety of ways, threatening human survival and development. Therefore, with the improvement of health awareness and the rapid development of science and technology, people are increasingly concerned about the development of products with bactericidal and antibacterial effects. Antibacterial means the process of inhibiting the growth and development of bacteria, thus reducing their performance. The process of killing bacteria to make the environment bacteria-free is sterilization. Currently, antibacterial materials refer to new materials with the function of inhibiting or killing microorganisms, and such bactericidal function is mainly achieved by adding antibacterial agents to materials [17].

There are great differences in the methods of preparing antibacterial textile materials at home and abroad. The domestic methods of preparing antibacterial textile materials include directly using antibacterial fibers to make various kinds of antibacterial textile materials, and the antibacterial properties of antibacterial textile materials are obtained by filling antibacterial agents and finishing. The methods of developing antibacterial fiber include the chemical starvation technique, adding antibacterial agent into spinning solution, physical modification technique, and compound spinning technique. Post-finishing processing methods include the microcapsule method, resin finishing method, and surface coating method [18].

The main methods for preparing antibacterial textile materials abroad include electroless plating, which is the deposition of thin films by chemical reaction between metal ions in solution and reducing agent. Vacuum evaporation deposition means that the basic material is first put into a vacuum box to achieve a vacuum environment. When the wire is heated to a certain temperature, evaporative deposition occurs, and the vaporized metal is deposited on the surface of the underlying material to form a coating. Magnetron sputtering method is to use the positive ions generated by the gas discharge point to bombard the target at a high speed under the action of electric field, so that the atoms in the target material escape and deposit to the surface of the plated basic material, thus forming the required film [19]. The main technical principles of magnetron sputtering are shown in Figure 2.

Magnetron sputtering is the current foreign advanced method of preparation of antibacterial textile materials, which has many advantages. This method allows the substrate to obtain a film of uniform thickness over a large area, and it can achieve any material sputtering basically. In addition, the combination between film and substrate fastness is strong, and it is quite friendly to the environment as well [20].

### 2.3. Research Design

The topic of the research is to investigate the application progress of ceramic nanofibers in antibacterial textile materials by CiteSpace software. CiteSpace is an information visualization software program, which was first launched in September 2004. After long-term updating and optimization, CiteSpace has become an important technical means for literature information visualization analysis. Literature retrieval using this software mainly includes four steps, which are subject determination, data retrieval, project setting, and mapping and interpretation [21]. The topic of the research is ceramic nanofibers and antibacterial textile materials. The version of CiteSpace is CiteSpace V5.8.R3c.  Figure 3 shows the main interface of CiteSpace.

As shown in Figure 3, CiteSpace can restrict search results by keyword, year, and author. The data sources searched in the research mainly include foreign and domestic sources. The foreign data source is Web of Science (WoS), which is an information retrieval platform maintained by a foreign company. WoS contains more than 8,000 peer-reviewed high-quality journals, which are among the most influential in the world. Also, scholars can access this database to search for research in different disciplines [22]. The data source in China is China National Knowledge Infrastructure (CNKI). CNKI project is an information construction project, which aims to spread knowledge resources to the whole society and promote the sharing and utilization efficiency of knowledge resources. It was founded by Tsinghua University and Tsinghua Tongfang in June 1999 [23].

## 3. The Evaluation of the Application of Ceramic Nanofibers Based on CiteSpace

### 3.1. The Evaluation of the Research on Ceramic Nanofibers

Based on CiteSpace software, the present situation of the application of ceramic nanofibers was investigated and evaluated. The main research object in the process of the investigation was ceramic nanofibers. Since the physical and chemical properties of ceramic nanofibers are very prominent, they are widely used in energy storage, electrochemical, photoelectric materials, environmental engineering, catalytic industry, and other fields.  Figure 4 shows the retrieval results of the research on the application of ceramic nanofibers.

As shown in Figure 4, OC refers to organic chemicals field. ICI refers to inorganic chemical industry. MS stands for material science, and PI stands for power industry. Retrieval results show that the number of Chinese literature is obviously lower than that of foreign literature. The number of Chinese literature is about 6,000 at most and 1,000 at least. The foreign literature is about 9,200 at most and about 6,300 at least.

### 3.2. The Evaluation of the Research on the Application of Ceramic Nanofibers in Antibacterial Textile Materials

Ceramic nanofibers are not only very light in weight and highly stable at high temperature but also have excellent mechanical strength and corrosion resistance, so it is a very wise choice to use them as antibacterial textile materials.  Figure 5 shows the evaluation results of the application of ceramic nanofibers in antibacterial textile materials in the research.

As shown in Figure 5, BS refers to biomedical science. The retrieval results show that the number of literature in Chinese is about 600 at most and 30 at least, indicating that the current domestic research on the application of ceramic nanofibers in antibacterial textile materials is not mature enough. In the foreign language retrieval, the number of documents is about 1,300, at least about 220, so it can be seen that the foreign language retrieval results are relatively good.

## 4. Conclusions

With the development of society, the quality of human life is constantly improving and people's pursuit of quality of life is also constantly rising. So, health has become an important indicator to ensure the quality of human life. Based on this, the antibacterial textile material application research is increasing. As a lightweight high-quality antibacterial material, ceramic nanofibers are considered an important substrate for antibacterial textile materials. Based on this, in the research, ceramic nanofibers were introduced firstly, then the principle and function of antibacterial textile materials were discussed, and finally the application of ceramic nanofibers in antibacterial textile materials based on CiteSpace software was investigated. The results show that the rise of ceramic nanofibers after 2000 is an important period. Since 2000, the number of Chinese literature is significantly lower than that of foreign literature. The number of Chinese literature was about 6,000 at most and 1,000 at least. The foreign literature was about 9,200 at most and about 6,300 at least. On the application of ceramic nanofibers in antibacterial textile materials, the number of literature in Chinese was about 600 at most, at least about 30, indicating that the application of ceramic nanofibers in antibacterial textile materials in China was not mature enough. In the foreign language retrieval, the number of documents was about 1,300, at least about 220, so it could be seen that the foreign language retrieval results were relatively good. It could be seen that the current research on ceramic nanofibers became mature, but its application in antibacterial textile materials is not mature enough. Although more accurate data are provided in the research, the keywords used in the research are not detailed enough. Therefore, in the future research, the refinement of keywords will be strengthened and the comprehensive application of ceramic nanofibers in antibacterial textile materials will be deeply investigated.

## Figures and Tables

**Figure 1:** The main design of the electrostatic spinning technology.

**Figure 2:** The main technical principle of magnetron sputtering method.

**Figure 3:** The main interface of CiteSpace.

**Figure 4:** Retrieval results of ceramic nanofibers: (a) in Chinese; (b) in foreign language.

**Figure 5:** Evaluation results of the application of ceramic nanofibers in antibacterial textile materials: (a) the Chinese retrieval result; (b) the foreign retrieval result.

**Table 1:** The main raw materials of ceramic nanofiber materials prepared by the electrostatic spinning technology.

Material classification	Material	Solvent name	Polymer carrier
(1) Metal oxide	Al_2_O_3_	C_2_H_5_OH	PVP
	CeO_2_	H_2_O	PVA
	Co_3_O_4_	DMF	PVP
	TiO_2_	C_2_H_5_OH	PVP
	CuO	H_2_O	PVA
	Fe_2_O_3_	H_2_O	PVA
	SiO_2_	H_2_O + C_2_H_5_OH	
	SnO_2_	H_2_O + C_3_H_7_OH + IPA	PVA
	ZrO_2_	C_2_H_5_OH	PVP
	V_2_O_5_	CHCl_3_ + DMF	PMMA
	WO_3_	C_3_H_7_OH + DMF	(C_4_H_6_O_2_)n
	BaTiO_3_	IPA	PVP
	CoFe_2_O_4_	DMF + THF	(C_4_H_6_O_2_)n
	NiO	H_2_O	
	MgTiO_3_	2-ME	PVAc
	ZnCo_2_O_4_	C_2_H_5_OH	PVP

(2) Metal nitride	VN	DMF	PVP
	TiN	C_2_H_5_OH + CH_3_COOH	PVP
	Li_3_N	H_2_O	PVA

(3) Metal carbide	Mo_2_C	H_2_O	PVA
	TiC	DMF	PVP
	ZrC	C_2_H_5_OH	PVP

## Data Availability

The data used to support the findings of this study are available from the corresponding author upon request.
